# Application Value of Metagenomics Next-Generation Sequencing (mNGS) in Detection of Mucormycosis after Chemotherapy in Childhood Acute Leukemia

This article has been retracted.

**DOI:** 10.1155/2022/7366432

**Published:** 2022-08-19

**Authors:** Wenzi Li, Hua Zhu, Li Wen, Meijie Quan, Li Wang

**Affiliations:** ^1^Department of Hematology and Oncology, Hebei Province Children's Hospital, Shijiazhuang City 050031, Hebei Province, China; ^2^Hebei Province Children's Hospital Orthopedics Department, Shijiazhuang City 050031, Hebei Province, China

## Abstract

**Objective:**

To analyze the application of macrogenomics next-generation sequencing (mNGS) in the detection of postchemotherapy trichomoniasis cases in children with acute leukemia.

**Methods:**

To retrospectively analyze the clinical data of 7 patients with acute leukemia combined with trichomoniasis after chemotherapy in the department of hematology and oncology of Hebei Children's Hospital, and to summarize the characteristics of their postchemotherapy clinical data, diagnostic and therapeutic processes, and outcomes.

**Results:**

Among the 7 children, 6 cases had acute lymphoblastic leukemia and 1 case had acute myeloid leukemia. mNGS detected trichoderma infection, including 1 case of pulmonary cerebral type and 6 cases of pulmonary type. After treatment, 1 case died, 2 cases were cured, and 4 cases improved.

**Conclusion:**

The clinical manifestations of trichomoniasis after combined chemotherapy in pediatric acute leukemia lack specificity. Early application of the mNGS assay is of great value.

## 1. Introduction

Pulmonary trichomycosis is an invasive pulmonary fungal disease caused by pathogenic infections of the order Trichophyton [1]. It occurs in immunocompromised populations, especially in immunodeficient hosts undergoing chemotherapy and hematopoietic stem cell transplantation [2]. Childhood acute leukemia is the most common hematologic malignancy in children[3]. The cure rate has gradually increased with the continuous improvement of chemotherapy regimens [4]. The combination of pulmonary trichomoniasis after chemotherapy can seriously affect the prognosis of children [5]. Because of the difficulty in treating this devastating infection, rapid initiation of antifungal therapy is the cornerstone [6]. However, the early diagnosis of pulmonary trichomycosis lacks specificity and relies mainly on histopathology and fungal culture, with long lead times and low positive rates [7]. In recent years, with the advent of mNGS assays, the detection rate of pathogenic organisms in children with postchemotherapy coinfection in leukemia has improved [8]. In this study, we retrospectively analyzed seven children with acute leukemia who had early infection detected by the mNGS method after chemotherapy for leukemia from January 2020 to December 2021, and analyzed the clinical characteristics, treatment, and outcome of these children [9]. The value of this method in the early diagnosis of pulmonary trichinosis after chemotherapy in children with acute leukemia was further discussed [10].

## 2. Cases and Methods

The clinical data of 7 children with acute leukemia complicated with mucormycosis treated in the Hematology and Oncology Department of Hebei Children's Hospital from 2020 to 1 to 2021–12 were collected. Mucormycosis was diagnosed in all 7 patients by the mNGS assay. There were 6 males and 1 female. The underlying diseases, clinical manifestations, laboratory and imaging examinations, use of antifungal drugs, surgical and other outcomes of 7 children were retrospectively analyzed. Reference (6) criteria for the evaluation of clinical efficacy: ① Cure: the symptoms and signs disappeared completely, and the lesions were obviously absorbed or completely absorbed by imaging examination; ② Improved: the symptoms and signs improved, and there was no significant change in the absorption of the lesions; ③ Worsening: new symptoms appeared. Symptoms and signs of infection, imaging examination progressed or did not improve; ④ death.

## 3. Results

### 3.1. Clinical Features

The clinical features of the 7 patients are shown in Table 1. Basic disease: 1 case of acute myeloid leukemia. The primary disease was not relieved when the infection occurred. During the second course of induction chemotherapy, the patient was in a state of agranulocytosis when the infection occurred, and the agranulocytosis lasted for 45 days. 6 cases of acute lymphoblastic leukemia, all patients achieved complete remission. During consolidation chemotherapy, they were in agranulocytosis state when infection occurred, and the duration of agranulocytosis was 8–18 days. All the children had been applied with more than two kinds of broad-spectrum antibiotics during hospitalization.

The time from symptom onset to diagnosis of pathogenic bacteria in 7 cases was 2–15 days, with an average of 7.85 days. Among the 7 cases of mucormycosis, 6 cases were of the pulmonary type, and they all showed varying degrees of fever and cough at the beginning of the disease, and the Case 4 showed rapid breathing. In 1 case of the pulmonary brain type, fever and cough were the first symptoms, followed by headache and convulsions.

### 3.2. Auxiliary Examination

7 children were in an agranulocytosis state during the course of the disease. The blood culture, sputum culture, sputum fungal smear, galactomannan (GM test) and 1,3 *β D* glucan (*G* test) were all negative. In Case 1, pathogenic bacteria were found through peripheral blood (PB) mNGS. The pathogenic bacteria were found in the PB and cerebrospinal fluid (CSF) mNGS of the lung-cerebral type (Case 2). In cases 4 and 5, pathogenic bacteria were found by mNGS of bronchoalveolar lavage fluid (BAL). In cases 3 and 6, pathogenic bacteria were found by mNGS in PB and BAL. In Case 7, pathogenic bacteria were found in the mNGS of PB but not found in the mNGS of BAL. Chest computed tomography (CT) manifestations of 6 children with pulmonary type were patchy shadow, nodular shadow, mass shadow, and consolidation. The cranial magnetic resonance (MRI) findings of a child with pulmonary cerebral type showed diffuse abnormal enhancement on the brain surface, sulci, and brain stem margins, as in Table 1.

### 3.3. Treatment and Outcome

All children were given liposomal amphotericin B formulation (LAmB) for injection and posaconazole oral liquid combined with antifungal therapy on the basis of controlling the primary disease. At the same time, amphotericin B was given by aerosol inhalation. The dose of amphotericin B liposome is 1–3 mg/kg·d. During the course of treatment, hypokalemia occurred in all 7 children. Renal function abnormalities occurred in 3 children, which improved after dose reduction or drug withdrawal. Cases 3, 5, 6, and 7 underwent bronchoalveolar lavage through fiberoptic bronchoscopy many times, but there was no significant improvement in repeated chest computed tomography scans. Case 6 underwent surgical resection of the diseased lung lobe due to lung consolidation and cavity formation. The postoperative pathological report was a fungal infection (Figures 1 and 2). Cases 1 and 7 were complicated with pulmonary hemorrhage due to severe cough during the follow-up consolidation chemotherapy. Case 1 improved after emergency surgery to remove the lesion, and Case 7 improved after timely invasive ventilator support. In Case 2, the condition of the child continued to progress, and during hospitalization, there were multiple convulsions, all of which were generalized seizures, and later the child died of multiple organ failure.

## 4. Discussion

Mucormycosis is a rare but extremely fatal invasive fungal disease. Several studies have shown that the underlying disease in patients is also related to the site of infection; pulmonary mucormycosis is more common in patients with hematologic malignancies and neutropenia, nasal orbital cerebral mucormycosis is more common in patients with diabetes, and trauma usually leads to cutaneous mucormycosis [11]. Pulmonary mucormycosis infection is one of the most common types of infections in patients with mucormycosis, and its nonspecific symptoms include fever, cough, dyspnea, and chest pain [12]. The lesions usually involve the lung parenchyma but may also extend to the chest wall, pulmonary artery, aorta, mediastinum, or pericardium, and hemoptysis may be caused by infiltration into the pulmonary artery [13]. In the present study, all children with mucormycosis were in a granulocytopenic state, including six cases of pulmonary mucormycosis and one case of pulmonary cerebral mucormycosis [14]. All patients had varying degrees of cough and fever at the beginning of the disease, and 2 patients developed hemoptysis during the progression of the disease.

Several studies have shown that the mortality rate of localized infections with mucormycosis is 20%–50%, while the mortality rate of disseminated mucormycosis can be as high as 70%–90% [15]. As treatment of this devastating infection is very difficult, rapid initiation of antifungal therapy is the cornerstone. Early diagnosis and treatment will help to reduce patient mortality. However, the diagnosis of mucormycosis depends on histopathology and culture. Mucormycosis readily invades blood vessels and destroys the tissue of affected organs, leading to vascular thrombosis and tissue necrosis with the formation of black crusts [16]. Hematoxylin-eosin (HE) staining, hyperoside (PAS) staining, and hexosamine silver staining can be selected for definite infection, with hexosamine silver staining being preferred, and may show broad, irregular hyphae in tissue specimen sections without separation or with little separation or righting branching [17]. In general, tissue cultures may be negative and blood cultures are rarely positive, even when there are characteristic histopathological changes of mucormycetes. Serological tests for galactomannan (GM test) and 1,3-beta-D glucan (G test) of mucor were negative [5]. In our study, blood cultures, sputum cultures, fungal smears in sputum, G and GM tests were negative in all children sent for examination. Only one case of resected diseased lung lobe was positive for hexosamine-silver staining, a characteristic change of mucormycosis infection, and no pathogenic evidence was found in other children by conventional laboratory tests [18].

In recent years, a new detection technology, metagenomic next-generation sequencing (mNGS), has emerged. mNGS does not require traditional microbial culture, does not require specific amplification, and can simultaneously detect known or unknown bacteria, fungi, viruses, parasites, and other pathogens in the same sample without bias [19]. The DNA or RNA in the sample is detected and then analyzed in comparison with the information database to know the species of pathogenic microorganisms contained in the sample [20]. Currently, mNGS has been gradually applied to the diagnosis of difficult clinical infections, and the types of specimens mainly include venous blood, cerebrospinal fluid, bronchoalveolar lavage fluid, sputum, pleural effusion, ascites, pharyngeal secretions, lesion punctures, and pathological tissues [21].

In our study, we used the mNGS assay to obtain evidence of pathogenic bacteria by infecting children with PB, BAL, and CSF. Four different mucus genera were identified [22]. In Case 2, the pathogenic bacteria were consistent in CSF and peripheral blood. Pathogenic bacteria in peripheral blood and alveolar lavage fluid were concordant in patients 3, 4, 5, and 6, respectively [23]. In all cases, it took only 1–2 days from specimen submission to report the test results. The time was greatly reduced. In combination with the test results, the treatment plan was rapidly adjusted and effective interventions were given, resulting in the survival of most of the children with a good prognosis [24].

## 5. Conclusion

The lack of specificity in the clinical manifestations of children with acute leukemia after chemotherapy makes it difficult to rely on clinical diagnosis at an early stage and to give effective interventions early, resulting in an extremely poor prognosis and high mortality. Therefore, early diagnosis and treatment are particularly important. mNGS is a novel detection technology that can shorten the time to detect pathogenic bacteria and can enable clinicians to give effective treatment plans in a timely manner, thus improving the prognosis of children, increasing their cure rate and reducing mortality. Therefore, mNGS detection technology is of great value in the early diagnosis of combined mucormycosis after chemotherapy for pediatric acute leukemia.

## Figures and Tables

**Figure 1:** Immunofluorescence of fungal hyphae.

**Figure 2:** Hexamine silver staining showed that the fungal hyphae were short black rod-like structures.

**Table 1:** Overview of our 7 pediatric mucormycosis cases.

Number	Age/sex	Underlying diseases	Main clinical manifestations	Specimen source/pathogenic bacteria/reads	Imaging performance	The involved organs	Antifungal drugs	Operative	Survival outcome
1	15/M	AML	Fever and cough	PB/Rhizopus mi Crosporus/(reads 125)	High-density shadow under the left lung	Lungs	LAmB posaconazole	Yes	Cure

2	11/F	ALL	Fever, cough, headache, and convulsions	PB/Rhizopus delemar/Reads 42 CSF/Rhizopus delemar/Reads 316	Cranial MRI: diffuse and abnormal enhancement on the brain surface, sulcus and brainstem margin chest CT: shadow of left lung	Lungs brain	LAmB posaconazole	No	Die

3	3/M	ALL	Fever and cough	PB/Rhizopus microsporus/reads 10 BAL/Rhizopus Microsporus/reads 10	High-density shadow in the lower lobe of both lungs	Lungs	LAmB posaconazole	No	Improved

4	1/M	ALL	Fever, cough breathe fast	BAL/Rhizomucor pusillus/reads 6	Real changes in the upper lobe of the left lung	Lungs	LAmB posaconazole	No	Improved

5	1/M	ALL	Fever, cough	BAL/Rhizomucor pusillus/Reads 3742	Double lung field multiple size unequal nodular sheet high-density shadow	Lungs	LAmB posaconazole	No	Improved

6	3/M	ALL	Fever cough	BAL/Rhizomucor pusillus/reads2 PB/Rhizomucor pusillus/reads 40	Large upper lobe of the right lung	Lungs	LAmB posaconazole	Yes	Cure

7	7/F	ALL	Fever cough	PB/Cunninghamella bertholletiae/reads 3	High-density shadow of emerging nodules in the lower lobe of the right lung	Lungs	LAmB posaconazole	No	Improved

ALL, acute lymphoblastic leukemia; AML, acute myeloid leukemia; CT, computerized tomography; MRI, magnetic resonance; PB, peripheral blood; BAL, bronchoalveolar lavage fluid; CSF, cerebral spinal fluid; LAmB, liposomal amphotericin B formulation.

## Data Availability

The experimental data used to support the findings of this study are available from the corresponding author upon request. The original contributions presented in the study are included in the article/supplementary materials. Further inquiries can be directed to the corresponding author.
